# The antagonism of 6-shogaol in high-glucose-activated NLRP3 inflammasome and consequent calcification of human artery smooth muscle cells

**DOI:** 10.1186/s13578-019-0372-1

**Published:** 2020-01-09

**Authors:** Te-Chuan Chen, Chia-Kung Yen, Ying-Chen Lu, Chung-Sheng Shi, Rong-Ze Hsieh, Shun-Fu Chang, Cheng-Nan Chen

**Affiliations:** 1 Division of Nephrology, Kaohsiung Chang Gung Memorial Hospital and Chang Gung University College of Medicine, Kaohsiung, Taiwan; 2 Department of Food Science, National Chiayi University, Chiayi, Taiwan; 3 Graduate Institute of Clinical Medical Sciences, College of Medicine, Chang-Gung University, Taoyuan, Taiwan; 4 Division of Colon and Rectal Surgery, Department of Surgery, Chang Gung Memorial Hospital, Chiayi, Taiwan; 5 Department of Medical Research and Development, Chang Gung Memorial Hospital, Chiayi, Taiwan; 6 Department of Biochemical Science and Technology, National Chiayi University, Chiayi, 600 Taiwan

**Keywords:** 6-Shogaol, Interleukin-1β, NLRP3 Inflammasome, Vascular calcification, Smooth muscle cells

## Abstract

**Background:**

Vascular calcification is the major reason for high mortality of cardiovascular complications for diabetes. Interleukin (IL)-1β has been implicated in this pathogenesis, but its precise role and clinical evidence have not been clearly identified. Hence, this study was aimed to investigate whether high concentration of glucose (HG), which mimics the hyperglycemia environment, could initiate vascular calcification through NLRP3/IL-1β inflammasome and the underlying mechanism. Recently, 6-shogaol, a major ginger derivate, has been elucidated its pharmaceutic role for various diseases. Therefore, the aims of this study also determined 6-shogaol effect in vascular calcification of HG initiation.

**Result:**

Human artery smooth muscle cells (HASMCs) were used in this study. Glucose concentrations at 5 and 25 mM were defined as normal and HG status, respectively. The results showed that HG could increase the NLRP3, cleaved caspase 1, and pro/mature IL-1β levels to induce the expressions of bone-related matrix proteins and subsequent HASMC calcification. This process was regulated by Akt activation and reactive oxygen species (ROS) production. Moreover, 6-shogaol could inhibit the Akt/ROS signaling and NLRP3/caspase 1/IL-1β inflammasome and hence attenuated HASMC calcification.

**Conclusions:**

This study elucidates the detailed mechanism of HG-initiated HASMC calcification through NLRP3/caspase 1/IL-1β inflammasome and indicates a potential therapeutic role of 6-shogaol in vascular calcification complication of diabetes.

## Background

Vascular calcification is highly prevalent for the patients with diabetes and chronic renal diseases and contributes to the further increased morbidity and mortality of cardiovascular complications. Although the therapeutic strategy for reducing blood glucose level has been extensively investigated, the vascular calcification development in diabetes patients have still remained [1–5]. Vascular calcification pathogenesis is a complex process with a phenotypic switch of vascular smooth muscle cells (VSMCs) to osteoblast- or chondrocyte-like cells, which initiates the upregulation and deposition of calcium phosphate and mineralization-related proteins, including osteopontin (OPN), osteocalcin (OCN), and alkaline phosphatase (ALP), in calcification regions and hence results in the stiffening of vessel walls [6–8]. Moreover, the signaling related to the bone/cartilage growth, including the bone morphogenetic proteins, Akt signaling, and runx2 transcription activity, has also been associated with the occurrence of vascular calcification complication of diabetes [8–12]. Currently, the precise mechanisms about how high blood glucose affects the vascular calcification pathogenesis in diabetes patients has not been completely elucidated. Therefore, more detailed investigation and understanding is still urgent and necessary for further improving the development of diabetes and its vascular calcification complications.

Vascular calcification derived from atherosclerosis and diabetes has been demonstrated to be a chronic inflammation event, which is regulated by inflammatory cytokines such as tumor necrosis factor (TNF)-α and interleukin (IL)-1β. Therefore, inflammasome system has recently been implicated in the pathogenesis of vascular calcification [13–15]. NLRP3 complex, which is composed of NLRP3 protein, adaptor protein ASC, and caspase 1, has been indicated as one of important inflammasomes because of its regulatory role in autoimmune and inflammation [16–18]. After receiving the stimulations, intracellular NLRP3 level upregulation and subsequent caspase 1 activation could cleave the pro-IL-1β and pro-IL-18 into mature and active IL-1β and IL-18 and then consequently elicit inflammatory responses and diseases development [16–18]. Accumulating data has indicated that inflammasomes, including NLRP3 complex, are the important regulatory systems for the development of chronic metabolic diseases. In this study, we further examine whether high concentration of glucose, mimics the hyperglycemia environment of diabetes patients, stimulates vascular calcification through the NLRP3 inflammasome system.

Ginger has been widely used as the flavoring agent and spice in the beverage and cooking in all over the world. Accumulating data has also demonstrated the pharmaceutic role of ginger in various diseases such as anti-cancer [19, 20], anti-arthritis [21, 22], anti-gastrointestinal disease [23, 24], anti-inflammation [25], anti-oxidation [26], and anti-atherosclerosis [27–29]. It has been found that the pharmaceutic function of ginger is elicited by the nature of its bioactive compounds, including gingerols and their dehydrated products, shogaols. Generally, shogaols have been suggested to be more effective than gingerols in attenuating the patients’ uncomfortable and status. And, 6-shogaol is the most dominant one [30]. However, the molecular mechanism and metabolic fate of shogaols, including 6-shogaol, in antagonizing and improving the status of these diseases have not been clearly identified. Therefore, the precise pharmaceutic effects and targets of 6-shogaol should be further elucidated and understood in order to more widely using it in the clinical application for various diseases therapy.

In this study, we investigated the role of NLRP3 inflammasome in vascular calcification in response to high glucose environment and the possible antagonized role of 6-shogaol in this process. We found that NLRP3, cleaved caspase 1, and pro/mature IL-1β proteins could be upregulated to initiate human artery SMC (HASMC) calcification under high concentration of glucose stimulation. Moreover, this NLRP3 inflammasome upregulation was resulted from the Akt activation and ROS production. Furthermore, we also demonstrated the antagonized role of 6-shogaol in NLRP3 inflammasome activation and subsequent HASMC calcification. Our findings provide new insights into the understanding of NLRP3 inflammasome-initiated HASMC calcification under high glucose stimulation and indicate a potential pharmaceutic role of 6-shogaol in cardiovascular complication of diabetes.

## Results

### High concentration of glucose (HG) initiates HASMC calcification

OPN, OCN, and ALP, the well-known bone matrix proteins, inductions have been recognized as the markers of vascular calcification. HASMCs were kept as the controls or were treated with 5 mM (normal concentration of glucose, NG) or 25 mM (high concentration of glucose, HG) glucose or 25 mM mannitol (M) for 3, 7, and 14 days and then the mRNA and protein expressions of OPN, OCN and ALP were examined. Cells treated with HG significantly induced the OPN, OCN, and ALP mRNA (Fig. 1a–c) and protein (Fig. 1d) expression within 3 days and persisted for 14 days in HASMCs compared to the controls and NG-/mannitol-treated cells. Moreover, we determined whether HG treatment initiates the HASMC calcification. Cells were kept as the controls or were treated with NG, mannitol, or HG for 14 days and then the HASMC calcification was examined. Cells treated with NG and mannitol had no effect on the HASMC calcification. However, cells treated with HG initiated an increase in HASMC calcification (Fig. 1e).

**Fig. 1:** HG initiates HASMC calcification. **a**–**d** HASMCs were kept as the controls or were treated with 5 mM (normal concentration of glucose, NG) or 25 mM (high concentration of glucose, HG) glucose or 25 mM mannitol (M) for 3, 7, and 14 days and then the mRNA **a**–**c** and protein **d** expressions of OPN, OCN and ALP were examined. **e** HASMCs were kept as the controls or were treated with NG, mannitol, or HG for 14 days and then the HASMC calcification was examined by ARS stain and were detected at 405 nm. Data in **a**–**c** and **e** are mean ± SEM from three independent experiments. Results in **d** are representative of three independent experiments with similar results and the bar graphs are mean ± SEM from three independent experiments. *P < 0.05 vs. control cells

### HG activates NLRP3 inflammasome to modulate HASMC calcification

Recently, NLRP3 inflammasome has been implicated in various diseases development. We determined whether NLRP3 inflammasome constituents, including NLRP3, caspase 1, and IL-1β, expressions could be upregulated in HASMCs in response to HG. HASMCs were kept as the controls or were treated with NG or HG for 12, 24, or 48 h and then the mRNA and protein expressions of NLRP3, caspase 1 (pro and cleaved form), and IL-1β (pro and mature form) were examined. Cells treated with HG significantly induced NLRP3 mRNA (Fig. 2a) and protein (Fig. 2b) expression within 12 h and persisted for 48 h in HASMCs compared to the controls and NG-treated cells. Moreover, HG also increased cleaved caspase 1 and pro/mature IL-1β protein expressions in HASMCs (Fig. 2b). Cells treated with NG had a partial effect on IL-1β protein expressions in HASMCs (Fig. 2b). Furthermore, cell pretreated with NLRP3 inflammasome inhibitor, MCC950, significantly inhibited OPN, OCN, and ALP mRNA expressions (Fig. 2c) and HASMC calcification (Fig. 2d) of HG induction.

**Fig. 2:** HG activates NLRP3 inflammasome to modulate HASMC calcification. HASMCs were kept as the controls or were treated with NG or HG for 12, 24, or 48 h or 14 days and then the mRNA **a** and protein **b** expressions of NLRP3, caspase 1 (pro and cleaved form), and IL-1β (pro and mature form), the mRNA expressions of OPN, OCN, and ALP **c**, and HASMC calcification **d** were examined. Data in **a** and **c**, **d** are mean ± SEM from three independent experiments. Results in **b** are representative of three independent experiments with similar results and the bar graphs are mean ± SEM from three independent experiments. *P < 0.05 vs. control cells. ^#^*P *< 0.05 vs. DMSO/HG-treated cells

### HG increases ROS level in HASMCs to trigger NLRP3 inflammasome and subsequent calcification

HASMCs were kept as the controls or were treated with NG, mannitol (M), or HG for 24 h and then the intracellular ROS level was examined. Cells treated with HG showed an increase in the ROS level in HASMCs compared to the controls and NG-/mannitol-treated cells (Fig. 3a). Cells were kept as the controls or were pretreated with DMSO or NAC, a ROS scavenger, for 1 h and then treated with HG for 2 (inflammasome protein expressions) and 14 (OPN/OCN/ALP mRNA expressions and calcification) days. HASMCs pretreated with NAC significantly downregulated HG-increased NLRP3, cleaved caspase 1, and pro/mature IL-1β protein (Fig. 3b) and OPN/OCN/ALP mRNA (Fig. 3c) expressions and HASMC calcification (Fig. 3d).

**Fig. 3:** HG increases ROS level in HASMCs to trigger NLRP3 inflammasome and subsequent calcification. **a** HASMCs were kept as the controls or were treated with NG, mannitol (M), or HG for 24 h and then the intracellular ROS level was examined. **b**, **c** HASMCs were kept as the controls or were pretreated with DMSO or NAC, a ROS scavenger, for 1 h and then treated with HG for 2 and 14 days. The NLRP3, caspase 1 (pro and cleaved form), and IL-1β (pro and mature form) protein expressions **b**, OPN, OCN, and ALP mRNA expressions **c** in HASMCs, and HASMC calcification **d** were examined. Data in **a** and **c**, **d** are mean ± SEM from three independent experiments. Results in **b** are representative of three independent experiments with similar results and the bar graphs are mean ± SEM from three independent experiments. *P < 0.05 vs. control cells. ^#^*P *< 0.05 vs. DMSO/HG-treated cells

### Akt signaling in HASMCs regulates HG-triggered ROS production, NLRP3 inflammasome and subsequent calcification

HASMCs were kept as the controls or were treated with NG, mannitol (M), or HG for 4 h and then the Akt phosphorylation was examined. Cells treated with HG significantly induced Akt phosphorylation in HASMCs compared to the control and NG-/mannitol-treated cells (Fig. 4a). Cells were kept as the controls or were pretreated with (i) DMSO or LY294008, an akt phosphorylation inhibitor, or (ii) pcDNA empty vector (EV) or dominant negative (dn)-Akt-expressed plasmid and then treated with HG for 1 (ROS production), 2 (inflammasome protein expressions) and 14 (OPN/OCN/ALP mRNA expressions and calcification) days. Akt activity inhibition in HASMCs by LY294008 or dn-Akt-expressed plasmid pretreatment significantly downregulated HG-increased NLRP3 and pro/mature IL-1β protein (Fig. 4b) and OPN/OCN/ALP mRNA (Fig. 4c) expressions, intracellular ROS production (Fig. 4c), and HASMC calcification (Fig. 4d).

**Fig. 4:** Akt signaling in HASMCs regulates HG-triggered ROS production, NLRP3 inflammasome and subsequent calcification. **a** HASMCs were kept as the controls or were treated with NG, mannitol (M), or HG for 4 h and then the Akt phosphorylation was examined. **b**–**d** HASMCs were kept as the controls or were pretreated with (i) DMSO or LY294008, an akt phosphorylation inhibitor, or (ii) pcDNA empty vector (EV) or dominant negative (dn)-Akt-expressed plasmid and then treated with HG for 2 and 14 days. The NLRP3 and IL-1β (pro and mature form) protein expressions **b**, ROS production **c**, and OPN, OCN, and ALP mRNA expressions **c** in HASMCs, and HASMC calcification **d** were examined. Results in **a**, **b** are representative of three independent experiments with similar results and the bar graphs are mean ± SEM from three independent experiments. Data in **c**, **d** are mean ± SEM from three independent experiments. *P < 0.05 vs. control cells. ^#^*P *< 0.05 vs. DMSO/ or EV/HG-treated cells

### 6-Shogaol attenuates HG-triggered Akt activation, ROS production, NLRP3 inflammasome, and calcification in HASMCs

Next, we examined whether 6-shogaol, a ginger derivate and a natural anti-inflammation factor, regulates HG effect on HASMC calcification. HASMCs were kept as the controls or were pretreated with ethanol or 6-shagaol and then treated with HG for 4 h (Akt phosphorylation) and 1 (ROS production), 2 (inflammasome protein expressions), and 14 (OPN/OCN/ALP mRNA expressions and calcification) days. It was shown that 6-shagaol significantly attenuates HG-increased Akt phosphorylation (Fig. 5a), intracellular ROS production (Fig. 5b), and NLRP3 and pro/mature IL-1β protein expressions (Fig. 5c) in HASMCs. Moreover, 6-shagaol also significantly attenuated HG-induced OPN/OCN/ALP mRNA expressions in HASMCs (Fig. 6a) and HASMC calcification (Fig. 6b).

**Fig. 5:** 6-Shogaol attenuates HG-triggered Akt activation, ROS production, and NLRP3 inflammasome in HASMCs. **a**, **b** HASMCs were kept as the controls or were pretreated with ethanol or 6-shagaol and then treated with HG for 4, 24, and 48 h. The Akt phosphorylation, ROS production, and NLRP3/IL-1β (pro and mature form) protein expressions in HASMCs were examined. Results in **a** and **c** are representative of three independent experiments with similar results and the bar graphs are mean ± SEM from three independent experiments. Data in **b** are mean ± SEM from three independent experiments. *P < 0.05 vs. control cells. ^#^*P *< 0.05 vs. EtOH/HG-treated cells

**Fig. 6:** 6-shogaol attenuates HG-triggered HASMC calcification. **a**, **b** HASMCs were kept as the controls or were pretreated with ethanol or 6-shagaol and then treated with HG for 14 days. The OPN, OCN, and ALP mRNA expressions in HASMCs **a** and HASMC calcification **b** were examined. Data in **a**, **b** are mean ± SEM from three independent experiments. *P < 0.05 vs. control cells. ^#^*P *< 0.05 vs. EtOH/HG-treated cells

## Discussion

This study has characterized the mechanisms whereby high glucose initiates HASMC calcification development through NLRP3 inflammasome and the antagonized role of ginger derivate, 6shogaol, in this process, as summarized in Fig. 7. The systematic experiments demonstrated that (i) HG initiates an osteogenic switch of HASMCs through upregulating the expressions of osteogenic matrix proteins, i.e., OPN, OCN, and ALP and the development of calcification. (ii) This calcification-initiating development in response to HG is regulated by Akt signaling, ROS production and subsequent NLRP3/caspase 1/IL-1β inflammasome activation. (iii) 6-shogaol effectively antagonizes the HG effect on NLRP3 inflammasome activation and consequent HASMC calcification. Our findings provide new insights into the regulatory mechanism of NLRP3 inflammasome in vascular calcification development under high glucose stimulation and suggest a potential nature product, 6-shogaol, in antagonizing this process.

**Fig. 7:** Schematic representation of signaling pathways regulating HG-triggered vascular calcification in HASMCs and the attenuated effect of 6-shogaol

Vascular calcification accompanies the development of atherosclerosis and diabetes and is associated with the mortality risk in patients with these two diseases [31]. Both atherosclerosis and diabetes have been recognized as the chronic and low-grade inflammation events and therefore the increased cytokines in blood has been indicated as an important initiator for diseases pathogenesis. Our present results indicated that HG could initiate the HASMC calcification development through upregulating the NLRP3/caspase 1/IL-1β inflammasome. Although IL-1β is one of well-demonstrated atherosclerosis- and diabetes-stimulating cytokines, its precise role and secretion mechanism in vascular calcification complication of diabetes have not been clearly detected [31]. In contrast, accumulating data has highlighted the importance and regulation of NLRP3 inflammasome activation and subsequent IL-1β secretion in hyperglycemia. For examples, (i) it has been indicated that NLRP3-knockdown mice which decrease the secreted level of IL-1β has an improved status for insulin resistance development [32, 33]; (ii) Stienstra et al. found that the inhibition of caspase 1 activity, which is involved in NLRP3 inflammasome system and could cleave the pro-IL-1β to mature form, affects the adipocyte differentiation and insulin sensitivity [34]; (iii) Maedler et al. demonstrated that high concentration of glucose could stimulate IL-1β secretion from the β-cells and hence elicit glucotoxicity in human pancreatic islets [35]; and (iv) Zhou et al. elucidated that high concentration of glucose could also upregulate the thioredoxin-interacting protein expression (one of NLRP3 binding proteins) to increase IL-1β level [32]. Taking all of these findings together, including ours, although it still has a limitation in the clinical evidence, we strongly indicated the indispensable role of IL-1β secreted from NLRP3 inflammasome-dependent system in vascular calcification development under high glucose environment.

In addition to being a pungent flavor, the pharmaceutic role of ginger has also been demonstrated for many years. 6-shogaol is the dominant constituent in ginger to contribute to uncomfortable release and ailment alleviation. It has been suggested that the anti-oxidation and anti-inflammation properties of 6-shogaol could effectively attenuate the status of metabolic and inflammatory diseases, including the cancer, arthritis, and atherosclerosis [19–29]. Our results found that 6-shogaol could attenuate HG-initiated HASMC calcification development. Moreover, this attenuation is elicited through attenuating the ROS production and subsequent NLRP3 inflammasome activation in HASMCs. Our data supported the idea that ginger and 6-shogaol contribute to the anti-oxidation and anti-inflammasome activities in disease therapy. Recent diabetic mice/rats (including type I and II models) studies have shown the beneficial effects of ginger or its derivates, including 6-shogaol, on homeostatic control of blood glucose and/or insulin [36–38]. Moreover, the clinical trials have also found the blood glucose-lowering potential of ginger in patients with type II diabetes [39]. Although the importance of ginger/6-shogaol in diabetes has already been found, their precise mechanism in blood glucose control and even more in vascular complications development have not been elucidated clearly. Our study has provided one of antagonized mechanisms of 6-shogaol in vascular calcification under high glucose condition and further supported the possibility of its clinical application in diabetes patients.

The aberrant activation of NLRP3 inflammasome has already been implicated in the pathogenesis of many diseases, including the diabetes. Therefore, targeting the NLRP3 inflammasome has been proposed as a promised method to improve these diseased. However, the therapeutic strategies specifically antagonizing the NLRP3 inflammasome have not been effectively developed and applied in patient treatment. The current study has reported that HG condition could result in vascular calcification through inducing the bone-related matrix protein, i.e., OPN, OCN, and ALP, expressions in HASMCs, which is regulated by the Akt activation, ROS production, and subsequent NLRP3/caspase 1/IL-1β inflammasome. Also, it has been further demonstrated that 6-shogaol, a nature ginger extract, could have an antagonized effect in HASMC calcification through inhibiting HG-activated NLRP3 inflammasome.

## Conclusion

The presented study provides new insights into understanding the mechanisms of NLRP3 inflammasome-regulated vascular calcification in HASMCs under hyperglycemia conditions. The results concerning the antagonized role of 6-shogaol might lead to the design and development of ginger-containing dietary therapy and/or new drugs for treating vascular calcification complication of diabetes through targeting the NLRP3 inflammasome.

## Methods

### Materials

Rabbit polyclonal antibody (pAb) against ALP and mouse monoclonal antibody (mAb) against OPN and OCN were purchased from Santa Cruz Biotechnology (Santa Cruz, CA). Rabbit pAbs against NLRP3, caspase 1, IL-1β, pAkt, Akt and β-actin were purchased from Cell Signaling Technology (Beverly, MA). Intracellular ROS assay kit was purchased from Cell Biolabs (San Diego, CA). MCC950 (NLRP3 inflammasome inhibitor), *N*-acetylcysteine (NAC, ROS inhibitor), and LY294002 (PI3K/Akt inhibitor) and other chemicals were purchased from Sigma (Temecula, CA).

### Cell culture

HASMCs were purchased from ATCC cell bank (Rockville, MD) and were cultured in medium (F12K, 10% FBS, and 1% antibiotics). Only 3–7 passages of HASMCs were employed for the experiments.

### HASMC calcification

SMC calcification is a mineralization process. It could be examined by Alizarin Red S (ARS) stain, a tool for detecting calcium deposition [40]. HG-treated HASMCs were fixed with formaldehyde (10%) and stained with ARS reagent (40 mM). Then, the stained HASMCs were extracted with acetic acid and then were neutralized with ammonium hydroxide. The samples were centrifugated and the supernatants were collected and measured at 405 nm by colorimetric detection.

### Quantitative real-time PCR

The cDNA extracted and converted from purified RNA of HASMCs was employed to determine the mRNA expression of the specific genes. The ABI StepOnePlus machine and SYBR Green kit (Applied Biosystems) were employed in the real-time PCR assay. The primers employed in the experiments included NLRP3 (positive: 5′- GATCTTCGCTGCGATCAACA-3′; negative: 5′- GGGATTCGAAACACGTGCATTA-3′), OPN (positive: 5′-GGACAGCCAGGACTCCATTG-3′; negative: 5′-TGTGGGGACAACTG GAGTGAA-3′), OCN (positive: 5′-GTGACGAGTTGGCTGACC-3′; negative: 5′-CAAGGG GAAGAGGAAAGAAGG-3′), ALP (positive: 5′-CTCCCAGTCTCATCTCCT-3′; negative: 5′-AAGACCTCAACTCCCCTGAA-3′) and GAPDH (positive: 5′-AGGTGAAGGTCGGAG TCAAC-3′; negative: 5′-CCATGTAGTTGAGGTCAATGAAGG-3′) genes. The GAPDH gene expression was indicated as the internal control.

### Western blot

HASMCs (controls and HG-treated) were lysed with lysis buffer (1% NP-40/0.1% SDS/0.5% sodium deoxycholate/protease and phosphatase inhibitor cocktail). The lysates (30 µg) were separated and examined by SDS-PAGE (10% running and 4% stacking) and the indicated antibodies.

### Plasmid transfection

HASMCs were cultured overnight and then transfected with the pcDNA empty vector or dominant negative Akt (dn-Akt)-expressed plasmids [41] by using the Lipofactamine 3000 Transfection Regents.

### Statistical analysis

The results were shown as mean ± SEM and the statistical analysis was measured by an independent Student t-test for two groups of data and analysis of variance (ANOVA) followed by Scheffe’s test for multiple comparisons. The *P* value < 0.05 was shown significant. Results were assayed from at least 3 repetitions which were collected from individual experiments.

## Data Availability

The data that support the findings of this study are available from the corresponding author upon reasonable request.

## Abbreviations

VASMCs: vascular artery smooth muscle cells
OPN: osteopontin
OCN: osteocalcin
ALP: alkaline phosphatase
IL-1β: interleukin-1β
pAb: rabbit polyclonal antibody
mAb: mouse monoclonal antibody
NAC: *N*-acetylcysteine
ARS: Alizarin Red S
dn-Akt: dominant negative Akt
HG: high concentration of glucose
NG: normal concentration of glucose
